This article has been retracted.

# Urinary Kallidinogenase plus rt-PA Intravenous Thrombolysis for Acute Ischemic Stroke: A Systematic Review and Meta-Analysis of Randomized Controlled Trials

**DOI:** 10.1155/2022/1500669

**Published:** 2022-05-17

**Authors:** Jing Wu, Jiang Wu, Le Wang, Jinmin Liu

**Affiliations:** ^1^Beijing University of Chinese Medicine, Beijing 100029, China; ^2^Dongfang Hospital Beijing University of Chinese Medicine, Beijing 100078, China

## Abstract

**Purpose:**

This research is aimed at systematically assessing the safety and effectiveness of intravenous thrombolysis (IVT) with rt-PA plus human urinary kallidinogenase (HUK) for acute ischemic stroke (AIS).

**Methods:**

The data were obtained through rigorous searching of both domestic and foreign databases from inception to 2021.7.1. Randomized controlled trials (RCTs) were included for the comparison of the efficacy of IVT plus HUK. The Cochrane risk of bias (RoB) tool and Review Manager software 5.3 were responsible for RoB assessment and statistical analyses, respectively.

**Results:**

A total of 18 articles were retrieved, including 2676 AIS patients treated with IVT within the time window. The control group used standardized rt-PA IVT, and the test group added HUK. After 14 days of combined application of HUK, the National Institute of Health Stroke Scale (NIHSS) score was significantly better in moderate stroke patients using the combination treatment versus those with IVT alone (mean difference (MD) = −3.13; 95% confidence intervals (CI): -3.40,-2.86; *P* < 0.00001); the NIHSS score was also statistically in severe stroke patients with combined treatment than in those with IVT alone, but the degree of recovery of patients varied greatly. After 90 days of treatment, the NIHSS (MD = −1.93; 95% CI: -2.51,-1.34; *P* < 0.00001) and Barthel index (BI) scores (MD = 22.23; 95% CI: 18.96, 25.49; *P* < 0.00001) of patients plus HUK were significantly better than those of patients with IVT alone, with fewer adverse events during treatment (Relative Risk (RR) = 0.66; 95% CI: 0.47, 0.92; *P* = 0.02).

**Conclusions:**

For AIS patients with IVT within the time window, HUK plus rt-PA IVT could significantly improve the neurological function recovery after 14 days and the quality of life after 90 days and reduce the adverse reactions of IVT. This trial is registered with CRD42021226975.

## 1. Introduction

Stroke is a prime reason for global adult death and disability [1], with AIS occupying 69.6%-70.8% of all stroke cases [2], seriously comprising people's health. The continuous advances in AIS treatment have substantially reduced patient mortality and improved the prognosis. Particularly, intravenous thrombolysis (IVT), endovascular therapy, and other reperfusion therapy have significant effects on patients [3].

For AIS patients meeting certain conditions, rt-PA IVT is a vital means for vascular recanalization recommended by national guidelines (level I recommend, level A evidence) [4]. However, in addition to the strict time window limitation, the clinical application of rt-PA still has the following problems to be solved: (1) in patients with thrombolytic rt-PA, only 10%-25% can achieve effective and permanent recalculation of occlusive vessels, because the drug half-life of rt-pa is only 5-10 minutes, which can hardly dissolve larger or older thrombus; (2) exogenous rt-PA can penetrate intact and damaged blood brain barrier (BBB) into ischemic brain tissue and produce neurotoxic effects; (3) rt-PA can increase BBB permeability and cerebral edema and induce cerebral hemorrhage; (4) after vascular recanalization, vascular reocclusion and reperfusion injury may occur [5, 6].

Tissue kallikrein (TKK) is a subgroup of acid glycoproteins highly consistent in gene and protein structures, and their sequences have great homology, colocalizing at the shared chromosomal loci 19q13.2-q13.4 [7]. Abundant in a variety of tissues, it has been confirmed to participate in multiple pathophysiological processes (e.g., inhibition of oxidative stress, apoptosis, and inflammation; promotion of angiogenesis, fibrosis, and neurogenesis) [8]. HUK, a member of TKK and can be separated from human urine, can activate the kallikrein-kinin system, convert kininogen into kinin, thereby increasing the plasma kinin level, expand small arteries in cerebral ischemic areas, and aggregate antiplatelet effects [9]. The medical value of HUK has been extensively studied, especially for the treatment of AIS [10].

At present, there are many clinical studies on the combined application of thrombolysis and HUK, but no one has conducted a comprehensive analysis of the efficacy and safety of the combination therapy. Therefore, this is the first meta-analysis of IVT alone in AIS and its combination with HUK to evaluate whether HUK has a synergistic effect on thrombolytic therapy and its adverse effects. The objective is to provide a basis for clinical application of HUK.

## 2. Methods

### 2.1. Inclusion and Exclusion Criteria for Studies

Inclusion criteria: (1) clinical randomized controlled study of IVT with rt-PA and HUK in patients with AIS, (2) thrombolytic therapy was standardized within the therapeutic time window (TTW) recommended by the guidelines [11], and HUK was administered intravenously.

Exclusion criteria: (1) patients who do not use rt-PA at the recommended dose or in the manner recommended by the guidelines; (2) used other treatments than those recommended by the guidelines.

### 2.2. Treatments

Control group: rt-PA IVT. Test group: HUK was administered intravenously at the same time as IVT or after thrombolytic therapy.

Additionally, the same basic interventions, including blood pressure control, oxygen inhalation, water-electrolyte balance maintenance, and intracranial pressure reduction, were carried out in both cohorts. Please see the Guidelines for the Early Management of Patients With Acute Stroke from the American Heart Association/American Stroke Association^4^ for details.

### 2.3. Primary Outcomes

The main endpoints included death and improvement of neurological impairment evaluated by clinical scales (e.g., NIHSS [12] and Glasgow outcome scale [13]).

### 2.4. Secondary Outcomes

The secondary evaluation indicators include (1) treatment response rate, including cure, obviously effective and effective rates, (2) life quality (e.g., European quality of life scale [14] and Barthel index [15]), (3) infarct area, and (4) peripheral blood biological indices.

### 2.5. Safety Outcomes

HUK-related adverse effects (AEs) included bleeding, hepatorenal function impairment, skin irritation, and nausea.

### 2.6. Literature Search Scope

The following databases were used to conduct electronic searches from the establishment of the database to 2021.7.1 with no language restriction: China National Knowledge Infrastructure (CNKI), SinoMed, WanFang Data, Chinese Science and Technology Periodical Database (VIP), PubMed, EMBASE, and Cochrane Library.

### 2.7. Keywords Searching

The keywords we used were stroke, cerebrovascular/cerebral/acute/acute ischaemic stroke, brain/cerebral infarction, cerebral/brain ischemia, cerebrovascular disorders, cerebral artery disease, cerebrovascular disease, cerebrovascular/brain vascular accident, apoplexy, cerebrovascular apoplexy, thrombolytic therapy, therapeutic thrombolysis, IVT, thrombolysis, thrombolytic, fibrinolytic therapy (therapies), urinary kallidinogenase, human tissue kallidinogenase, urinary kallikrein, kallikrein, urinary kallid, HUK, human urinary kallidinogenase, and tissue kallikrein. According to each database's characteristics, keyword searching was carried out using the method of combining subject words and free words. The detailed PubMed search strategy is shown in Table 1.

### 2.8. Data Acquisition and Processing

Literature screening and information acquisition were carried out by 2 researchers independently after reading the related literature. The following information was obtained: (1) general article information: author names and publication materials; (2) patient data: mean age, case number, gender; (3) HUK intervention: drug dosage, treatment duration; (4) treatment outcomes: response rate, activities of daily living, melioration of neurological impairment, complications, AEs during treatment, and mortality. The consistency of the data extracted were double checked by researchers. Any discrepancy was settled through negotiation or jointly decided by a third-party researcher.

### 2.9. Risk of Bias (RoB) Assessment

Following the RCT RoB evaluation criteria of the Cochrane Systematic Review *v*5.2, the two researchers conducted independent assessment regarding literature quality, taking into the account the bias of random sequence generation, allocation concealment, blinding (research subjects and personnel, and outcome assessment), selective outcome reporting, and incomplete outcome data. Each item was rated as either low, high or unclear risk. Any disagreement was settled by consultation.

## 3. Statistical Processing

Review Manager software 5.3 was responsible for statistical processing. We used relative risk (RR) to evaluate binary variables' effect sizes, and used mean difference (MD) as continuous variables' efficacy analysis statistics. For the presentation of interval estimation, 95% confidence interval was utilized. The results were analyzed by the random-effects model. The statistical heterogeneity of literature included was judged *P* and *I*^2^, with *P* > 0.1 + *I*^2^ < 50% and *P* < 0.1 + *I*^2^ ≥ 50% indicating small and high heterogeneity, respectively.

## 4. Results

### 4.1. Literature Retrieval Results

A comprehensive search of 7 databases with a total of 269 documents, including 21 in English and 248 in Chinese. Removing 166 duplicate documents, we further ruled out 4 animal experiments and 11 nonclinical treatment trials after read the title and abstract of the literature. By reading the full text, we continued to screen out 35 articles against the inclusion criteria and 4 not according with the standard of curative effect evaluation, 16 non-RCT, 7 thrombolysis outside the TTW, 7 documents with incomplete data, and 1 repeated publication, eventually included 18 documents. See Figure 1 for the screening flowchart.

### 4.2. Features of Included Literature

Eighteen RCTs comprising 2676 patients (male-to-female ratio: 1.29 : 1) [16–33] were eventually selected, all of whom were AIS patients receiving thrombolytic therapy within 6 hours of onset. Among the included literature, 17 [17–33] were in Chinese, and 1 [16] was in English, published between 2015 and 2020. All studies were dual-arm trials, with one group receiving intravenous rt-PA thrombolysis and the other receiving HUK on the basis of thrombolysis. All studies exhibited no statistically significant difference in baseline data between groups. A summary of the baseline data, treatment medications, and outcome indicators included in the literature is shown in Table 2.

Among the 18 RCTs, 11 reported the method of random grouping [17, 20, 21, 23–25, 28, 29, 31–33], all of which was random number table method, random sequence generation was evaluated as low risk, and other random methods were evaluated as unclear risk. Allocation concealment scheme, blind method of researcher or subject, and blind evaluation of research outcome were not reported in all literature. Therefore, allocation concealment, performance, and detection biases were all determined to be unclear risks. There was no missing data in all the studies, and the outcome evaluation was consistent with the scheme design without selective reporting. Therefore, both attrition bias and reporting bias are low risks. All the studies reported consistent baseline and comparability between the two groups of patients, so other bias was evaluated as low risk. The summary of Rob's studies is shown in Figure 2.

### 4.3. NIHSS Score on the 14th Day

NIHSS scores were recorded after 14 days of treatment in 8 studies, all of which were treated with HUK for 14 days. The results of the 8 studies were highly heterogeneous, so the severity of patients' disease was assessed according to the average NIHSS score at the time of inclusion, and subgroup analysis was conducted. At the time of enrollment, 5 < NIHSS < 15 was considered as a moderate stroke, and NIHSS ≥ 15 was considered as a severe stroke.

5 studies [21, 22, 25, 30, 31] included patients with moderate stroke, and the results showed obviously better neurological recovery in patients with combined HUK after 14 days of treatment compared with those with IVT (MD = −3.13; 95% CI: -3.40,-2.86; *P* < 0.00001), without any heterogeneity among the 5 articles (*P* = 0.21, *I*^2^ = 32%). The results of 3 studies [20, 27, 33] involving patients with severe stroke also showed that the combined application of HUK is better than simple IVT, but the heterogeneity between the 3 studies is large, analysis of sources of heterogeneity, it may be that the patient's recovery is not only affected by treatment, besides factors such as the severity of the disease at the time of onset and the patient's chronic have a greater impact on the outcome. When patients are seriously ill and receive the same treatment, their clinical outcomes will still vary greatly (Figure 3).

### 4.4. NIHSS Score on the 90th Day

4 studies [16, 17, 19, 28] recorded the 90-day NIHSS score of patients, and the results showed better neurological recovery in patients with combined HUK versus those with IVT (MD = −1.93; 95% CI: -2.51,-1.34; *P* < 0.00001), without heterogeneity among the 4 papers (*P* = 0.14, *I*^2^ = 46%) (Figure 4).

### 4.5. BI Score on the 90th Day

6 studies [16–19, 22, 28] recorded the 90-day BI score of patients, and the results showed that the 90-day clinical prognosis of patients with combined HUK was significantly better than that of IVT patients (MD = 22.23; 95% CI: 18.96, 25.49; *P* < 0.00001), without any heterogeneity among the six papers (*P* = 0.14, *I*^2^ = 39%) (Figure 5).

### 4.6. AEs and Publication Bias

12 studies [17, 20, 22–26, 28, 29, 31–33] documented the AEs of treatments, including cerebral hemorrhage, gastrointestinal hemorrhage, gum bleeding, urinary tract hemorrhage and hypotension, chest tightness, nausea, and vomiting. The results showed a lower incidence of AEs under the combined application of HUK compared with IVT alone (RR = 0.66; 95% CI: 0.47, 0.92; *P* = 0.02), without heterogeneity in 12 studies (*P* = 0.17, *I*^2^ = 29%) (Figure 6(a)).

The assessment of publication bias used a funnel plot, and 12 articles documenting patients' AEs were evaluated. Both sides of the inverted funnel plot are symmetrical, and the dots represented by all studies are within the range of oblique lines on both sides of the 95% confidence interval, indicating that there is no publication bias in the included studies. For the sensitivity analysis, removing any of the 12 included studies did not affect the comparison of results (Figure 6(b)).

### 4.7. Death and Other Indicators

2 studies [18, 26] recorded the death of patients 90 days after the onset of the disease, and 1 study [18] recorded the patient's recurrence of cerebral infarction within 1 year. The results determined no evident difference between groups (*P* > 0.05).

In the included literature, a variety of indicators were also used to evaluate the effect of drug treatment, such as the TCD breath-hold test was used to detect the hemodynamics of the main arteries and the physiological parameters of the blood flow on the intracranial base of the arterial ring. Various indicators are vascular endothelial growth factor (VEGF) and hypersensitive C-reactive protein (hs-CRP) levels before and after. Due to the inconsistent observation indicators of various studies, statistical analysis cannot be combined. However, individual studies have demonstrated the significant therapeutic effect of the combined application of HUK.

## 5. Discussion

### 5.1. Summary of Results

This study, as far as we know, is the first comprehensive review regarding the postthrombolysis application value of HUK, and the included studies are the results of data published in the past 6 years. This study included 18 prospective randomized controlled studies, including 2676 AIS patients undergoing thrombolysis within the TTW. The control group used standardized rt-PA IVT and basic interventions recommended by the guidelines, and the test group added HUK. The NIHSS score is a series of measurements of neurological deficits in patients [12]. It divides neurological functions into 11 categories with a total score of 42 points. The more serious neurological deficits are, the higher the score is, and the normal people without neurological deficits is 0 point.

The NIHSS score was used as the most important criterion for evaluating the efficacy in this study, and with a 15-point boundary, the degree of neurological deficit at the onset of the patients was divided into moderate and severe. Significantly better NIHSS scores were found in moderate stroke patients treated with combined application of HUK 14 days after treatment, as compared to those with IVT alone; the NIHSS score of patients with severe stroke was also significantly better, but the degree of recovery of patients varied greatly. The results showed that the combination of HUK could significantly reduce NIHSS scores and improve the neurological deficits of moderate and severe patients after 14 days of onset. After 90 days of treatment, the NIHSS and BI scores of patients combined with HUK were significantly better than those of patients with IVT alone, and the number of AEs during treatment was statistically lower.

The results of our study are the first to comprehensively analyze the therapeutic effect of HUK on IVT patients, confirm the clinical value of the combined application of HUK, and provide evidence for clinicians to use HUK.

### 5.2. Feasibility Mechanism

In recent years, great progress has been made in both intravenous thrombolysis and endovascular thrombectomy [34], which has significantly improved the functional independence of patients, especially allowing for thrombolytic therapy in patients who are after awakening and with unknown onset time under conditions of MRI-DWI positive and FLAIR negative [35]. However, it is pressing to solve the problems of the recanalization rate and complications of thrombolysis. Exploring an effective combined application that can improve the efficacy of IVT and reduce its AEs has always been a clinical challenge.

HUK is a research hotspot with extensive clinical application as it shows favorable curative effects. The effectiveness of HUK for AIS has been demonstrated in recent clinical trials and animal experiments. On the one hand, in HUK-intervened patients, enhanced microcirculation and cerebral hemodynamics were observed, which may facilitate neurogenesis and angiogenesis, and suppress inflammation and apoptosis [10]. The effectiveness of HUK for AIS was studied based on the TOAST classification, and it was found that HUK validly improved the NIHSS score of large- and small-artery atherosclerosis-induced cerebral ischemia [36]. HUK treatment resulted in markedly enhanced cerebral blood perfusion in AIS patients, and shortened mean perfusion transit time, which explains the increase in serum contents of VEGF and apelin [37], both of which participate in blood vessel formation and maturation [38]. On the other hand, HUK was capable of promoting neurogenesis and angiogenesis postischemia/reperfusion (I/R) injury, as demonstrated by animal experiments [39]. Continuous infusion of hypotensive doses of HUK through micropumps can reduce I/R-induced neurological disorders, cerebral infarction, inflammation, as well as oxidative stress, indicating the antioxidative and antiinflammatory action of HUK that can protect the brain against AIS damage [40].

### 5.3. Limitations

(1) Although both English and Chinese were included, all clinical studies were conducted in China, which may affect the judgment and extrapolation of the outcome. (2) The 18 included studies are generally low-quality studies with a higher risk of overall methodological deviation, and they are all small-sample studies, and the experimental scheme also needs to be optimized. (3) The treatment period of HUK included in the study varies in length, of the 18 studies, 12 treatments lasted for 14 days, while others included 7, 21, and 30 days. The number of included studies was too small to conduct subgroup analysis. (4) Among the included literature, only 2 articles recorded death of the patient within 90 days. Therefore, the safety of warrants further investigation.

### 5.4. Implication for Clinical Practice

In future clinical trials, many measures can be improved: (1) in clinical medication, although the treatment course of HUK is less than one month, the short-term effect at the end of the treatment course can be recorded, and the long-term curative effect can be carried out. Follow-up to observe the long-term prognosis of the drug on patients. (2) Make detailed records of the generative process of the random sequence, the allocation concealment scheme, and the implementation of the blind method. According to the research purpose and research type, a scientific and rational sample size estimation is conducted. All these can improve the quality of the literature and increase the credibility of the literature.

## 6. Conclusions

According to meta-analysis, for AIS patients with IVT within the TTW, HUK plus IVT could significantly improve the neurological function recovery after 14 days and the quality of life after 90 days and reduce the adverse reactions of IVT. Therefore, clinicians can add HUK to IVT patients according to their wishes based on the results of our study to promote better recovery. However, due to the small sample size and low quality of the included studies, the research on HUK is still in its preliminary stage, and large randomized controlled trials with strict protocol design and standardized reports are needed to explore the best treatment regimen for HUK, as well as its effectiveness and safety for the long-term prognosis of patients.

## Figures and Tables

**Figure 1:** Flowchart of literature screening.

**Figure 2:** Proportion of offset risk results.

**Figure 3:** Forest plot with NIHSS score on the 14th day.

**Figure 4:** Forest plot with NIHSS score on the 90th day.

**Figure 5:** Forest plot with BI score on the 90th day.

**Figure 6:** (a) Forest plot of adverse effects; (b) funnel plot of documents publication.

**Table 1:** Search strategy for the PubMed database.

Number	Search items
#1	“Stroke”[mesh]
#2	((((((((((((((cerebrovascular stroke[title/abstract])OR(cerebral stroke[title/abstract]))OR (acute stroke[title/abstract]))OR(acute ischaemic stroke[title/abstract]))OR(brain ischemia[title/abstract]))OR(brain infarction[title/abstract]))OR(cerebral infarction[title/abstract])) OR (cerebral ischemia[title/abstract])) OR (cerebrovascular disorders[title/abstract])) OR (cerebrovascular disease[title/abstract]))OR(cerebrovascular accident[title/abstract])) OR (cerebralartery disease[title/abstract]))OR(brain vascular accident[title/abstract]))OR (apoplexy[title/abstract])) OR (cerebrovascular apoplexy[title/abstract])
#3	#1 OR #2
#4	“Thrombolytic therapy”[mesh]
#5	(((((Intravenous thrombolysis[title/abstract]) OR (thrombolysis[title/abstract])) OR (thrombolytic[title/abstract])) OR (fibrinolytic therapy[title/abstract])) OR (fibrinolytic therapies[title/abstract])) OR (therapeutic thrombolyses[title/abstract])
#6	# 4OR #5
#7	“Tissue plasminogen activator”[mesh]
#8	(((tPA[title/abstract]) OR (rtPA[title/abstract])) OR (alteplase[title/abstract])) OR (T plasminogen activator[title/abstract])
#9	#7 OR #8
#10	“Tissue kallikreins “[mesh]
#11	(((((Urinary kallidinogenase[title/abstract]) OR (human tissue kallidinogenase[title/abstract])) OR (urinary kallikrein[title/abstract])) OR (kallikrein[title/abstract]))OR (HUK[title/abstract])) OR (human urinary kallidinogenase[title/abstract])
#12	#10 OR #11
#13	#3 AND #6 AND # 9 AND #12

**Table 2:** Characteristics of selected clinical trials included in the meta-analysis.

Study ID	Sample size (T/C)	Sex (M/F)	Age	HUK dosage	Course	Outcomes	AEs (T/C)
Wang YX2015	100/100	109/91	T: 58.8 ± 10.6 C: 61.2 ± 9.7	0.15PNA	7 d	②③	Unclear
Du CY2017	30/30	38/22	T: 62.08 ± 2.75 C: 61.47 ± 3.02	0.15PNA	14 d	②③	Unclear
Gong LY2019	83/80	87/76	T: 69.6 ± 8.5 C: 68.7 ± 7.0	0.15PNA	14 d	③	3/2
Gu WY2016	100/100	102/98	T: 60.2 ± 9.8 C: 61.3 ± 9.4	0.15PNA	7 d	②③	Unclear
Gu YL2018	65/65	69/61	T: 55.08 ± 1.1 C: 54.91 ± 1.23	0.15PNA	14 d	①	4/4
Huang YW2018	54/54	57/51	T: 4.91 ± 1.23 C: 62.58 ± 5.24	0.15PNA	14 d	①	Unclear
Jiang TL2018	45/45	53/37	T: 55.1 ± 13.0 C: 60.2 ± 12.7	0.15PNA	14 d	①③	3/3
Jiang B2017	51/51	60/42	T: 57.64 ± 5.21 C: 56.23 ± 5.08	0.15PNA	30 d	④	5/6
Li HT2020	57/57	57/57	T: 68.8 ± 2.9 C: 69.2 ± 3.2	0.15PNA	14 d	④	2/8
Li H2020	43/43	53/33	T: 55.25 ± 6.01 C: 54.61 ± 5.96	0.15PNA	14 d	①	3/12
Lv ZY2017	207/219	262/164	T: 64.2 ± 12.7 C: 63.4 ± 12.5	0.15PNA	7 d	④	65/80
Ma XL2020	69/69	79/59	T: 53.0 ± 1.5 C: 52.8 ± 1.4	0.15PNA	14 d	①	Unclear
Tong CM2020	57/57	62/52	T: 55.37 ± 5.11 C: 54.97 ± 5.05	0.15PNA	21 d	②③	5/6
Wang W2016	38/38	41/35	T: 55.23 ± 14.37 C: 56.37 ± 13.92	0.15PNA	7 d	④	6/18
Yao ZG2018	200/200	224/176	T: 61.93 ± 12.45 C: 62.15 ± 12.37	0.15PNA	10~14 d	①	Unclear
Yu YL2020	36/36	45/27	T: 64.23 ± 3.16 C: 64.45 ± 3.27	0.15PNA	14 d	①	None
Zhao FH2018	59/58	68/49	T: 62.1 ± 6.0 C: 62.0 ± 6.0	0.15PNA	14 d	④	5/13
Zhuang X2020	40/40	43/37	T: 64.44 ± 3.10 C: 64.24 ± 3.22	0.15PNA	14 d	①	9/8

Note: T: test group; C: control group; outcomes: (1) 14 d NIHSS; (2) 90 d NIHSS; (3): 90 d BI; (4) 7/30 d NIHSS; AEs: adverse events.

## Data Availability

The simulation experiment data used to support the findings of this study are available from the corresponding author upon request.
